# Seismic Random Noise Denoising Using Mini-Batch Multivariate Variational Mode Decomposition

**DOI:** 10.1155/2022/2132732

**Published:** 2022-02-26

**Authors:** Guoning Wu, Guochang Liu, Junxian Wang, Pingping Fan

**Affiliations:** ^1^College of Science, China University of Petroleum (Beijing), Beijing, China; ^2^State Key Laboratory of Petroleum Resources and Prospecting, China University of Petroleum (Beijing), Beijing, China

## Abstract

Seismic noise attenuation plays an important role in seismic interpretation. The empirical mode decomposition, synchrosqueezing wavelet transform, variational mode decomposition, etc., are often applied trace by trace. Multivariate empirical mode decomposition, multivariate synchrosqueezing wavelet transform, and multivariate variational mode decomposition were proposed for lateral continuity consideration. Due to large input data, mini-batch multivariate variational mode decomposition is proposed in this paper. The proposed method takes advantages both of variational mode decomposition and multivariate variational mode decomposition. This proposed method firstly segments the input data into a series of smaller ones with no overlapping and then applies multivariate variational mode decomposition to these smaller ones. High frequency-domain noise is filtered through sifting. Finally, the denoised smaller ones are concatenated to form components (or intrinsic mode functions) of the input signal. Synthetic and field data experiments validate the proposed method with different batch sizes and achieve higher signal-to-noise ratio than the variational mode decomposition method.

## 1. Introduction

Seismic noise attenuation plays an important role in seismic interpretation [1–3]. A variety of methods have been proposed for attenuating or removing random noise in order to enhance the signal-to-noise ratio (SNR) [4–8]. The transform-based methods, such as Fourier transform [9], wavelet transform [10], curvelet transform [11], and seislet transform [12], assume that the input signal has sparse representation with predetermined base, and under the predetermined base, noise and clean signal can be separated in the transform domain [7, 13–15].

Apart from these fixed basis methods mentioned above, there are also some data-driven methods [16]. Empirical mode decomposition (EMD) [17–19] recursively decomposes an input signal into so-called intrinsic mode functions (IMF); these IMFs are amplitude and frequency modulated subsignals with slow variations. EMD is widely used for trend detection and spectrum analysis in conjunction with Hilbert transform. Lack of a rigorous theory background for the EMD method leaves room for other decomposition methods to come. Synchrosqueezing wavelet transform (SWT) [20], a hybrid of wavelet transform and reassignment method, squeezes values of wavelet transform to its ridges in order to sharpen the time-frequency distribution. Another data-driven method is a nonparametric one called singular spectrum analysis (SSA) [21], which firstly computes the singular value decomposition of a covariance matrix derived from the input signal. After that, SSA decomposes the input signal into a sum of components with meaningful interpretations. SSA captures the basic periodicity of an input signal and is widely used in different areas [22]. Variational mode decomposition (VMD) [23] utilizes the alternative direction method of multipliers (ADMM) and nonrecursively decomposes an input signal into some principal modes. Like EMD and SSA methods, the decomposed modes of the VMD method are narrow banded and compact around some center frequencies.

Denoising methods based on EMD, VMD, and SSA, except in f-x fashion, are often applied trace by trace; lateral continuity is not considered [24–26]. In order to improve SNR, the multichannel spatial coherence needs to be considered. Multivariate empirical mode decomposition (MEMD) [27] and multivariate synchrosqueezing wavelet transform (MSWT) [28], as extensions of EMD and SWT, have been proposed to try to separate multivariate modes of faster oscillations from slower ones as a whole. Recently, multivariate variational mode decomposition (MVMD) [29], an extension of VMD, has emerged to seek a collection of multivariate modulated components with minimum collective bandwidth and full signal reconstruction property. These extended methods have been used in wide areas with multivariate data analysis, such as EEG and ECG applications [30–32]. With their effectiveness of these multivariate methods, they usually companied with high computational complexity due to large input data. Furthermore, it is a tricky problem for the parameters' setting. In view of these situations above, mini-batch multivariate variational mode decomposition (MB-MVMD) is proposed in this paper. The proposed method firstly segments the input data into a number of batches of fixed size with no overlapping. After that, it applies VMD or MVMD for the segmented data, depending on the input data which are segmented trace by trace or not. Noise on high-frequency domain is filtered through the sifting process. Finally, the decomposed data are concatenated to form components (or IMFs) of the input signal. The proposed method has the following advantages:

- VMD and MVMD are two special cases of the proposed method.
- Initial parameters can be set differently depending on different batch sizes.
- Lateral continuity is considered if the data are not segmented trace by trace.
- Instead of directly decomposing the input data as a whole, the MB-MVMD method segments the input signal into a series of smaller ones. Solutions to the smaller ones are then combined to give a solution to the original problem. This divide-and-conquer technique, therefore, promotes the computing efficiency.

## 2. From Univariate to Mini-Batch Multivariate Variational Mode Decomposition

### 2.1. Univariate Variational Mode Decomposition

The univariate variational mode decomposition seeks *K* number of intrinsic mode functions *u*_*k*_(*t*) such that

(1) $$\begin{array}{c} x\left(t\right)=\sum_{k=1}^{K}u_{k}\left(t\right), \end{array}$$

where *u*_*k*_(*t*)=*a*_*k*_(*t*)cos  *ϕ*_*k*_(*t*). These modes *u*_*k*_ are chosen to minimize the bandwidths sum and fully reconstruct the input signal *x*(*t*); these can be mathematically written as [23]

(2) $$\begin{array}{c} \underset{\left\{u_{k}\right\}\left\{\omega_{k}\right\}}{\min}\sum_{k=1}^{K}{\left\|\partial_{t}\left[u_{k}^{+}\left(t\right)e^{-j\omega_{k}t}\right]\right\|}_{2}^{2},\\ \text{s.t.}\;\sum_{k=1}^{K}u_{k}\left(t\right)=x\left(t\right), \end{array}$$

where {*ω*_*k*_} denotes the center frequency and *u*_*k*_^+^(*t*) denotes the analytic signal corresponding to *u*_*k*_(*t*):

(3) $$\begin{array}{c} u_{k}^{+}\left(t\right)=u_{k}\left(t\right)+jℋu_{k}\left(t\right), \end{array}$$

where ℋ denotes the Hilbert transform:

(4) $$\begin{array}{c} ℋu\left(t\right)=\frac{1}{\pi }\int_{-\infty }^{+\infty }\frac{u\left(t\right)}{t-x}\text{d}x. \end{array}$$

Equation (2) uses frequency modulation and Wiener filtering techniques.

For gratified solutions, two constraints are added to optimization (2) to form a Lagrangian problem:

(5) $$\begin{array}{c} ℒ\left(\left\{u_{k}\right\},\left\{\omega_{k}\right\},\lambda \right)=\frac{\alpha }{2}\sum_{k=1}^{K}{\left\|\partial_{t}\left[u_{k}^{+}\left(t\right)e^{-j\omega_{k}t}\right]\right\|}_{2}^{2}\\ +{\left\|x\left(t\right)-\sum_{k=1}^{K}u_{k}\left(t\right)\right\|}_{2}^{2}+\langle \lambda \left(t\right),x\left(t\right)-\sum_{k=1}^{K}u_{k}\left(t\right)\rangle . \end{array}$$

Alternative direction method of multipliers (ADMM) [23], summarized in algorithm (1), is used for the solution of optimization (5) in time domain.

For computational simplicity, the ADMM algorithm for VMD in time domain is transformed to frequency domain and is summarized in algorithm (2).

VMD nonrecursively decomposes input signal into modes with compacted bandwidths and limited amplitudes' variations. Since VMD decomposes input signal trace by trace, lateral continuity is not considered.

### 2.2. Multivariate Variational Mode Decomposition

Suppose the input signal consists of *M* channels, that is, **x**(*t*)=[*x*_1_(*t*), *x*_2_(*t*),…, *x*_*M*_(*t*)]. As an extension of the VMD method, we try to find *K* multivariate modulated components {**u**_*k*_(*t*)}_*k*=1_^*K*^ that will fully construct the input signal **x**(*t*):

(6) $$\begin{array}{c} x\left(t\right)=\sum_{k=1}^{K}u_{k}\left(t\right), \end{array}$$

where the *k*th multivariate component **u**_*k*_(*t*) is a vector with *M* components:

(7) $$\begin{array}{c} u_{k}\left(t\right)=\left[\begin{array}{c} u_{k,1}\left(t\right)\\ u_{k,2}\left(t\right)\\ \vdots \\ u_{k,M}\left(t\right) \end{array}\right]=\left[\begin{array}{c} a_{k,1}\left(t\right)\cos\left(\phi_{k,1}\left(t\right)\right)\\ a_{k,2}\left(t\right)\cos\left(\phi_{k,2}\left(t\right)\right)\\ \vdots \\ a_{k,M}\left(t\right)\cos\left(\phi_{k,M}\left(t\right)\right) \end{array}\right]. \end{array}$$

Let **u**_*k*_^+^(*t*) denote the Hilbert transform of **u**_*k*_(*t*):

(8) $$\begin{array}{c} u_{k}^{+}\left(t\right)=\left[\begin{array}{c} u_{k,1}^{+}\left(t\right)\\ u_{k,2}^{+}\left(t\right)\\ \vdots \\ u_{k,M}^{+}\left(t\right) \end{array}\right]=\left[\begin{array}{c} u_{k,1}\left(t\right)+jℋu_{k,1}\left(t\right)\\ u_{k,2}\left(t\right)+jℋu_{k,2}\left(t\right)\\ \vdots \\ u_{k,M}\left(t\right)+jℋu_{k,M}\left(t\right) \end{array}\right]=\left[\begin{array}{c} a_{k,1}\left(t\right)\exp\left(j\phi_{k,1}\left(t\right)\right)\\ a_{k,2}\left(t\right)\exp\left(j\phi_{k,2}\left(t\right)\right)\\ \vdots \\ a_{k,M}\left(t\right)\exp\left(j\phi_{k,M}\left(t\right)\right) \end{array}\right]. \end{array}$$

We modulate the *k*th multivariate component **u**_*k*_(*t*) by *ω*_*k*_; corresponding to equation (2), the constrained optimization problem for MVMD is

(9) $$\begin{array}{c} \underset{\left\{u_{k,i}\right\},\left\{\omega_{k}\right\}}{\text{argmin}}\sum_{k=1}^{K}\sum_{i=1}^{M}{\left\|\partial_{t}\left[u_{k,i}^{+}\left(t\right)e^{-j\omega_{k}t}\right]\right\|}_{2}^{2},\\ \text{s.t.}\;\sum_{k=1}^{K}u_{k,i}\left(t\right)=x_{i}\left(t\right),\;i=1,2,\ldots ,M. \end{array}$$

The Lagrangian function with added two constraints is

(10) $$\begin{array}{c} ℒ\left(\left\{u_{k,i}\right\},\left\{\omega_{k}\right\},\lambda_{i}\right)=\frac{\alpha }{2}\sum_{k=1}^{K}\sum_{i=1}^{M}{\left\|\partial_{t}\left[u_{k,i}^{+}\left(t\right)e^{-j\omega_{k}t}\right]\right\|}_{2}^{2}\\ +\sum_{i=1}^{M}{\left\|x_{i}\left(t\right)-\sum_{k=1}^{K}u_{k,i}\left(t\right)\right\|}_{2}^{2}+\sum_{i=1}^{M}\langle \lambda_{i}\left(t\right),x_{i}\left(t\right)-\sum_{k=1}^{K}u_{k,i}\left(t\right)\rangle . \end{array}$$

Just like algorithm (1), ADMM algorithm [29] is used for the solution of equation (10) in time domain and is summarized in algorithm (3).

ADMM algorithm [29] for MVMD in frequency domain is summarized in algorithm (4); it is simpler than MVMD in time domain.

MVMD takes multivariate input signal as a whole and tries to seek K number of multivariate components from the input signal with minimum sum of bandwidths. With big data input, ADMM for MVDM in frequency domain may have high computation complexity.

### 2.3. Mini-Batch Multivariate Variational Mode Decomposition

Mini-batch multivariate variational mode decomposition (MB-MVMD) takes the advantages of both VMD and MVMD methods. MB-MVMD segments the input data into a series of smaller ones with no overlapping; after the segmentation, these smaller ones are decomposed using ADMM method just as the MVMD or VMD. This mini-batch technique not only considers lateral continuity of the input data but also promotes the computational efficiency using divided-and-conquer technique.

Suppose the input data are **X** with *N* traces (or columns). We firstly set the batch size and then compute the number of batches using floor function “ ⌊⌋”:

(11) $$\begin{array}{c} \text{Number of batches}=\left\lfloor \frac{N}{\text{Batch size}}\right\rfloor . \end{array}$$

After that, we extract the *l*th mini-batch data from the input data **X**:

(12) $$\begin{array}{c} x_{l}=X\left[\left(l-1\right)*\left(\text{bs}\right):l*\left(\text{bs}\right)\right], \end{array}$$

where “bs” denotes the batch size previously determined. Following the segmentation above, we use ADMM algorithm in frequency domain to decompose the *l*th mini-batch data and lastly concatenate the decomposed data to form components.

The computation processes of MB-MVMD in frequency domain are summarized in algorithm (5).

## 3. Experimental Results

Figure 1 shows a single seismic trace and its four extracted components using the VMD method. These four components are narrow banded.  Figure 2 shows the sum of the four extracted components in Figure 1 and the difference between the sum and the original input single seismic trace. From these figures, we see that VMD extracts sub signals with compacted bandwidth subject to full signal reconstruction. The parameters for VMD decomposition are number of components *K* = 4 and bandwidth constraint *α*=500.

A bivariate signal with three different tones and a certain percentage of Gaussian noise is shown in Figure 3. We apply MVMD to this signal; the extracted components are shown in Figure 4(a). The parameters for the MVMD method are number of components *K* = 4 and bandwidth constraint *α*=500. For comparison, the MEMD method is also used to decompose this bivariate signal; results are shown in Figure 4(b). From these figures, we see that MVMD uses fewer components than the MEMD method to represent the input signal.

SNR is often used as a qualitative indicator to show the effectiveness of a denoising method; it is defined as the ratio of signal power to the noise power and is often expressed in decibels:

(13) $$\begin{array}{c} \text{SNR}=20\log_{10}\left[\frac{A_{s}}{A_{n}}\right], \end{array}$$

where *A*_*s*_ and *A*_*n*_ represent signal and noise powers.

### 3.1. Synthetic Data

A synthetic seismic data with four linear events are used for test. The synthetic data have 256 traces, with time step Δ*t*=0.004 and 512 samples. Figures 5(a), 5(b), and 5(c) are the synthetic signal, the random Gaussian noise, and the noisy data, respectively.  Figure 6 shows denoised results using three different methods: FX-DECON, VMD, and MB-MVMD. Figures 6(a), 6(b), and 6(c) show the denoised result, removed noise using FX-DECON, and the similarity between them. Figures 6(d), 6(e), and 6(f) show the denoised result, removed noise using VMD, and the similarity between them. The parameters of the VMD method are bandwidth constraint *α*=2000 and *τ*=0.0 and number of components *K* = 4. Figures 6(g), 6(h), and 6(i) show the denoised result, removed noise using MB-MVMD of batch size eight, and the similarity between them. The parameters of the MB-MVMD method are *α*=1000, *τ*=0.5, and*K*=4. From these figures, we can see that the denoised data of FX-DECON is better than the denoised one of VMD. The denoised data of MB-MVMD of batch size eight are the best, which can be seen from the denoised results, the removed noises, and the similarities of these three methods.

Another synthetic mode (shown in Figure 7) is used to test the proposed method. Figures 8(a), 8(b), and 8(c) are the denoised data, removed noise using FX-DECON, and similarity between them. Figures 8(d), 8(e), and 8(f) are the denoised data, removed noise using VMD, and similarity between them. Figures 8(g), 8(h), and 8(i) are the denoised data, removed noise using MB-MVMD of batch size four, and similarity between them. The parameters of the VMD method are bandwidth constraint *α*=2000and*τ*=0.0and number of components *K*=4. Parameters for MB-MVMD of batch size four are *α*=1000, *τ*=0.5,  and *K*=4. The denoised result of FX-DECON is better than the denoised result of VMD; the denoised data of MB-MVMD are the best among these three denoising methods. The MB-MVDM method considers the lateral continuity of the input data; some degree of signal is removed as noise, which can be seen from the removed noise data. Similarity of MB-MVDM of batch size four also reveals the effectiveness of the proposed method in random noise attenuation.

Table 1 shows the SNRs of the above two models using different batch sizes (Model 1 is the linear synthetic model and Model 2 is the synthetic model of Figure 7). The results show that the SNR of batch size eight is best for model 1, and the SNR of batch size four is best for model 2.

### 3.2. Field Data

Figure 9 shows a marine data; the data have 470 traces. Figures 9(a), 9(b), and 9(c) are the clean field data, Gaussian random noise, and the noisy data, respectively.

FX-DECON, VMD, and MB-MVMD of batch size five are used to denoise the noisy data. Figures 10(a), 10(b), and 10(c) are the denoised data, the removed noise using FX-DECON, and the similarity between them. Figures 10(d), 10(e), and 10(f) are the denoised data, the removed noise using VMD, and the similarity between them. Figures 10(g), 10(h), and 10(i) are the denoised data, the removed noise using MB-MVMD of batch size five, and the similarity between them. The removed noises show that a lot of signals are removed from the data for the VMD method, which is confirmed by the similarity of the VMD method (the “Signal” boxes indicate signal is removed as noise.). The removed signal as noise is least for the MV-MVMD method, which is also confirmed by the similarity of the MV-MVMD method.

Table 2 shows the SNRs of the three models using different denosing methods. “Model 1” is the synthetic model with linear events, “Model 2” is the second model, and “Field Data” is the field data model. The SNRs reveal that the MV-MVMD method is the best with respect to denoising results.

## 4. Conclusion

MB-MVMD considers the lateral continuity of the input data; it seeks a sparse representation of the input signal. This divide-and-conquer method bridges VMD and MMVD methods. The proposed method achieves better denoising results compared with the VMD method in seismic random noise denoising.

Although the proposed method has many advantages, there is still room for improvement. For example, the decomposition parameters are set manually; is there a way to automatically select the best parameters for the decomposition?

## Figures and Tables

**Figure 1:** VMD decomposition. From the top to bottom are the input signal and its VMD decomposition components.

**Figure 2:** Seismic trace and its sum of VMD components: “Original” is the input seismic signal, “Fit” is the sum of VMD components in Figure 1, and “Difference” is the difference between the input signal and its VMD approximation.

**Figure 3:** Bivariate signal: each has three components and a certain percentage of Gaussian noise. (a) The bottom of left column consists of three different tones (the top three signals in left column) and a certain percentage of Gaussian noise (the fourth signal in left column). (b) The bottom of right column also consists of three different tones and a certain percentage of Gaussian noise.

**Figure 4:** Decomposition of the bivariate signal in Figure 3. (a) MVMD: three components. (b) EMD: six components.

**Figure 5:** Synthetic seismic data with four linear events. (a) Clean data. (b) Gaussian random noise. (c) Data with noise added.

**Figure 6:** Denoise comparisons. (a) Denoised data using FX-DECON. (b) Removed noise using FX-DECON. (c) Similarity between denoised data and its removed noise using FX-DECON. (d) Denoised data using VMD. (e) Removed noise using VMD. (f) Similarity between denoised data and its removed noise using VMD. (g) Denoised data using MB-MVMD of batch size eight. (h) Removed noise using MB-MVMD of batch size eight. (i) Similarity between denoised data and its removed noised using MB-MVMD of batch size eight.

**Figure 7:** Synthetic seismic data with Gaussian noise. (a) Clean data. (b) Gaussian random noise. (c) Data with noise added.

**Figure 8:** Denoise comparisons. (a) Denoised data using FX-DECON. (b) Removed noise using FX-DECON. (c) Similarity between denoised data and its removed noise using FX-DECON. (d) Denoised data using VMD. (e) Removed noise using VMD. (f) Similarity between denoised data and its removed noise using VMD. (g) Denoised data using MB-MVMD of batch size four. (h) Removed noise using MB-MVMD of batch size four. (i) Similarity between denoised data and its removed noised using MB-MVMD of batch size four.

**Figure 9:** Field data with Gaussian noise. (a) Field data. (b) Gaussian random noise. (c) Field data with noise added.

**Figure 10:** Denoise comparisons. (a) Denoised data using FX-DECON. (b) Removed noise using FX-DECON. (c) Similarity between denoised data and its removed noise using FX-DECON. (d) Denoised data using VMD. (e) Removed noise using VMD. (f) Similarity between denoised data and its removed noise using VMD. (g) Denoised data using MB-MVMD of batch size four. (h) Removed noise using MB-MVMD of batch size four. (i) Similarity between denoised data and its removed noised using MB-MVMD of batch size four.

**Algorithm 1:** ADMM for VMD in time domain.

**Algorithm 2:** ADMM for VMD in frequency domain.

**Algorithm 3:** ADMM for MVMD in time domain.

**Algorithm 4:** ADMM for MVMD in frequency domain.

**Algorithm 5:** ADMM for MB-MVMD in frequency domain.

**Table 1:** SNRs (in decibels) comparison using different batch sizes.

Batch size	2	4	8	16	32	64	128	256
Model 1	4.78	4.81	**6.89**	6.55	6.43	6.10	5.97	5.43
Model 2	5.89	**6.27**	6.12	5.83	5.74	5.61	5.57	4.98

**Table 2:** SNRs' (in decibels) comparison using FX-DECON, VMD, and MB-MVMD.

	FX-DECON	VMD	MB-MVMD
Model 1 (linear events)	4.78	−0.94	6.89
Model 2 (synthetic data)	1.81	1.25	6.27
Field data	5.90	−1.87	7.35

## Data Availability

The data are not freely available due to third-party rights.
